# Toll-like receptor sensing of human herpesvirus infection

**DOI:** 10.3389/fcimb.2012.00122

**Published:** 2012-10-08

**Authors:** John A. West, Sean M. Gregory, Blossom Damania

**Affiliations:** ^1^Lineberger Comprehensive Cancer Center, University of North Carolina at Chapel HillChapel Hill, NC, USA; ^2^Department of Microbiology and Immunology, University of North Carolina at Chapel HillChapel Hill, NC, USA; ^3^UNC Center for AIDS Research, University of North Carolina at Chapel HillChapel Hill, NC, USA

**Keywords:** TLR, herpesvirus, innate immunity, cytokines, interferons

## Abstract

Toll-like receptors (TLRs) are evolutionarily conserved pathogen sensors that constitute the first line of defense in the human immune system. Herpesviruses are prevalent throughout the world and cause significant disease in the human population. Sensing of herpesviruses via TLRs has only been documented in the last 10 years and our understanding of the relationship between these sentinels of the immune system and herpesvirus infection has already provided great insight into how the host cell responds to viral infection. This report will summarize the activation and modulation of TLR signaling in the context of human herpesvirus infections.

## Introduction

Pathogen detection is critical in the establishment of an immune response by the host innate immune system. Recognition of microbial pathogens is primarily carried out by cell surface or endosomal receptors, which trigger signaling cascades that result in the upregulation of inflammatory cytokines and type I interferon (IFN) (Akira and Sato, 2003; Akira and Takeda, 2004). One of the key innate immune receptors, Toll receptors, was first identified in *Drosophila Melanogaster* as being responsible for detection of fungal infection. Subsequently, eleven homologs of the *Drosophila* Toll receptors have been identified in humans and are classified as Toll-like receptors (TLRs) (Akira et al., 2001). TLRs represent the first line of defense in the human innate immune response and consequently have become an intense focus of study in the response to virus infection. Understanding the role of TLRs during pathogen infection and the signaling events that occur in response to stimulation of TLRs helps to provide a clearer picture of the establishment of the innate immune response to viral infection.

TLRs are termed pattern recognition receptors (PRRs), a general name for a family of receptors capable of recognizing a wide variety of pathogen associated molecular patterns (PAMPs) (Slack et al., 2000). PAMPs are motifs common to large numbers of pathogens, which upon detection by TLRs leads to initiation of TLR signaling cascades, launching the host immune response (Akira and Hemmi, 2003). TLRs are type I membrane proteins that recognize their ligands via leucine rich repeat (LRR) motifs contained within their Ig-like ectodomains (Slack et al., 2000; Akira and Hemmi, 2003; Akira and Sato, 2003). Currently, eleven mammalian TLRs have been identified, however, only nine have been well characterized. TLR expression is cell type dependent and most cells express at least a small complement of TLRs. The location of TLRs in the cell aids in their ability to recognize a wide variety of invading pathogens. TLRs 1, 2, 4, 5, and 6 sense pathogens at the cell surface, while TLRs 3, 7, 8, and 9 are located on endosomal membranes and serve primarily as nucleic acid sensors (Akira et al., 2001; Akira and Sato, 2003; Akira and Takeda, 2004). This review will focus on the activation of TLR signaling in response to human herpesviruses infection.

The agonists have been identified for nine of the eleven mammalian TLRs, including each of the endosomal TLRs. TLR3 senses double-stranded RNA, a common intermediate in virus infection. Human TLR7 and TLR8 appear to have redundant functions, and recognize single-stranded RNA, another common intermediate during viral infection (Akira et al., 2001; Alexopoulou et al., 2001; Akira and Hemmi, 2003; Kariko et al., 2004a,b; Sarkar et al., 2004, 2007; Sen and Sarkar, 2005; Carpentier et al., 2007). TLR9 has been shown to bind CpG unmethylated DNA, a common sequence motif in DNA viruses but a relatively rare sequence in vertebrates (Hemmi et al., 2000; Bauer et al., 2001; Akira and Hemmi, 2003).

TLR signaling is mediated through one of two adapter proteins, MyD88 or TRIF. All TLRs, with the exception of TLR3 and one arm of the TLR4 pathway, initiate signaling via MyD88. TLR3 signals through the adapter protein TRIF (Kawai and Akira, 2006). TLR4 is capable of signaling through both MyD88 dependent and independent pathways (Kawai et al., 2001). Activation of the TLR response results in a signaling cascade generated to suppress and eradicate the invading pathogen. Increased production of inflammatory cytokines such as IL-6, type I IFN, a key component of the anti-viral state, and secretion of chemokines to attract innate immune cells, including neutrophils and macrophages, are all consequences of TLR activation (Akira and Takeda, 2004). Figure 1 summarizes human herpesvirus activation of TLR signaling. Herpesviruses are well known for their ability to control the host immune response in order to achieve latency (Damania, 2004; Melroe et al., 2004; Paladino and Mossman, 2009; Paludan et al., 2011). Therefore, activation of TLR signaling is often countered by the virus using viral encoded suppressors of host immune proteins, some targeted specifically to TLR signaling pathways. For each of the viruses discussed in this review we will also highlight viral proteins known to inhibit different aspects of TLR signaling.

**Figure 1:** **Human herpesviruses can stimulate a wide variety of TLRs leading to upregulation of both inflammatory cytokines and type I interferon. (A)** Activation of NF-κB and inflammatory cytokines (IL-6, IL-8, and IL-12) via TLR stimulation by human herpesviruses. TLR stimulation results in activation of NF-κB in the cytoplasm and subsequent translocation to the nucleus where it serves as a transcriptional activator for a large number of inflammatory cytokines. Activation of these cytokines can occur after stimulation of both endosomal and cell surface TLRs by human herpesviruses. **(B)** Activation of type I interferon in response to recognition of human herpesviruses by TLRs. Both IFN-α and IFN-β are activated by cellular interferon regulatory factors (IRFs), specifically IRF3 and IRF7, which translocate to the nucleus following phosphorylation and activate the IFN-α and IFN-β promoters. Activation of type I interferon are induced after stimulation of both cell surface TLRs (TLR2 and TLR4), and endosomal TLRs (TLR3, 7, and 9).

## α-Herpesviruses

### Herpes simplex virus—types 1 & 2

Human herpesviruses 1 and 2, more commonly known as herpes simplex types 1 and 2 (HSV-1 and HSV-2) are present in approximately 80% of the human population (Cunningham et al., 2006). Initial infection occurs either on the skin or in the oral or genital mucosa. Latent infection is established in cell bodies of neurons where the virus permanently resides in the host. HSV-1 infection can result in ocular herpes (which can lead to blindness), genital herpes, and encephalitis (most common in young children) (Cunningham et al., 2006). HSV-2 infection is the leading cause of genital herpes, which can lead to neonatal herpes, and infection with HSV-2 increases the likelihood of acquiring HIV almost 3 fold (Wald and Link, 2002; Cunningham et al., 2006).

Cytokine production as a result of TLR stimulation typically leads to virus clearance or aids in the control of viral spread via establishment of an anti-viral state through activation of IFN and recruitment of innate and adaptive immune cells to the site of infection. However, in some cases the release of cytokines following virus infection can have a detrimental effect on the host. In 2004, Kurt-Jones et al. reported that HEK293 cells constitutively expressing TLR2 showed increased IL-6 production in response to primary HSV-1 infection, and that this increase could be attributed to activation of NF-κB (Kurt-Jones et al., 2004). This report went on to demonstrate that while TLR2 does play an important role in recognition of HSV-1, it also contributes to encephalitis in infected mice. Wild type mice, TLR2^−/−^, and TLR4^−/−^ mice were challenged with equivalent amounts of HSV-1 via intraperitoneal injection. Significantly fewer mice succumbed to infection from the TLR2^−/−^ group and symptoms of disease were also reduced in TLR2^−/−^ mice compared to both wild type and TLR4^−/−^ mice, serum levels of IL-6 were significantly reduced in TLR2^−/−^ mice (Kurt-Jones et al., 2004). Because neonates are extremely susceptible to HSV-1 infection, neonatal mice were also challenged with HSV-1 and monitored for disease progression and symptoms. By day 6 post-infection, 90% of the wild type and TLR4^−/−^ mice had succumbed to infection, while over 60% of the TLR2^−/−^ mice survived and half of the survivors were symptom free throughout the study (Kurt-Jones et al., 2004). *The authors attributed the survival of TLR2^−/−^ mice to the reduction in cytokine levels and accompanying inflammation in the brain of the infected animals*.

The inflammatory responses among the different mouse groups varied drastically and indicated that TLR2-mediated cytokine responses to HSV-1 infection can be lethal in mice (Kurt-Jones et al., 2004). Elevated levels of IL-6 and *CCL2* were detected in the serum and brain, respectively, compared to the levels in wild type and TLR4^−/−^ mice. Inflammatory lesions were also observed in the brains of infected wild type and TLR4^−/−^ mice, but not in the brains of TLR2^−/−^ mice, despite similar virus titers in the brain (Kurt-Jones et al., 2004). This report suggests that the host response may contribute to the pathogenesis of HSV-1 infection, as much or sometimes more so than the virus infection itself.

A role for an additional TLR, TLR9, was also identified in HSV-1 infection of mice (Krug et al., 2004). Initially, CD11c^+^ splenocytes from wild type and MyD88 deficient mice were infected with HSV-1 via corneal infection and levels of IFN-α and IL-12 were measured. Both IFN-α and IL-12 levels were reduced in MyD88 deficient mice compared to wild-type controls. Plasmacytoid dendritic cells (pDCs) were then sorted from the CD11c^+^ population from both wild type and MyD88^−/−^ mice and were exposed to HSV-1. IFN-α and IL-12 levels were significantly increased compared to wild type controls (Krug et al., 2004). To determine whether TLR9 was responsible for the cytokine upregulation, pDCs were isolated from TLR9^−/−^ mice and infected with HSV-1. pDCs from TLR9 deficient mice displayed significantly less IFN-α activation along with reduced levels of IL-12 secretion. pDCs from TLR9^−/−^ mice also showed reduced levels of the activation marker CD86 compared to wild type controls. To confirm the specificity for TLR9, pDCs were infected in the presence of a TLR9 competitive inhibitor (ODN, 2088). In the presence of the inhibitor, HSV-1 infected pDCs from wild type animals showed lower levels of IFN-α and IL-12 and also reduced expression of CD86 (Krug et al., 2004) indicating that the recognition of HSV-1 is specific for TLR9 in murine pDCs.

Because HSV-1 resides in neurons during latency, cells within the brain that can mediate immune responses are key in controlling HSV infection and spread. Microglial cells are the macrophages of the brain; they sense invading pathogens and are critical in mounting proper immune responses within the brain (Aravalli et al., 2005). HSV infection of primary microglial cells isolated from wild type and TLR2^−/−^ mice revealed that TLR2 activation by HSV was required for the secretion of a wide variety of cytokines and chemokines including, IL-6, IL-12, CCLl7, CCL8, CCL9, CXCL1, CXCL2, CXCL4, CXCL5, IL-1β, and TNF-α (Aravalli et al., 2005).

HSV-1 infection can result in corneal keratitis following infection of the epithelial and stromal layers of the cornea (Li et al., 2005). It has been determined using human corneal epithelial cells, both immortalized cells (HUCL) and primary cells (HCECs), that TLR7 is induced upon HSV-1 infection while TLR3 is down regulated (Li et al., 2005). Infection of human corneal epithelial cells resulted in activation of multiple transcription factors including NF-κB, JNK, and p38 (Li et al., 2005). Activation of each of these factors occurred in two distinct peaks, first at 1–4 h post-infection and again at 8 h post-infection. Each peak could be further differentiated based on activation of a unique set of secondary factors. During the first peak activation (1–4 h), upregulation of several cytokines was also observed including IL-6, IL-8, TNF-α, and IFN-β. Concomitant with the second peak of activation (8 h), two significant changes in TLR expression were observed (Li et al., 2005). TLR7 levels were increased and TLR3 levels were decreased. The authors concluded that sequential regulation of these two TLRs was necessary for a proper immune response in epithelial cells.

In 2006, it was discovered that subpopulations of the KOS strain of HSV-1 and two strains of HSV-2, WT186 (186-K) and unique long region 29-deficient 186 strain (UL29^−^186-K), could activate TLR2 signaling based on NF-κB reporter assays. Activation of TLR2 also led to increased secretion of both IL-6 and IL-12 (Sato et al., 2006). This study also showed that activation of TLR9 by these subpopulations of HSV-1 and HSV-2 could occur in the same cell that had already recognized these incoming pathogens via TLR2. The activation of TLRs was sequential and the results suggested a new mechanism by which an invading pathogen could trigger TLR signaling via two distinct TLR pathways within the same cell (Sato et al., 2006).

There are conflicting reports in the literature about the activation of TLR2 by HSV-1 viral glycoproteins. It was initially reported that HSV-1 entry glycoproteins could be recognized by monocyte derived dendritic cells (Reske et al., 2008). Recognition of gB, gD, and gH/gL resulted in upregulation of CD40, CD83, CD86, IL-10, and IFN-α in these cells, however, the observed changes in each of these downstream inflammatory proteins was not dependent on binding of these viral glycoproteins to surface expressed TLR2 (Reske et al., 2008). However, a more recent report suggests that gB and gH/gL are both capable of binding TLR2 and that a soluble form of the gH/gL complex alone is sufficient to induce upregulation of NF-κB (Leoni et al., 2012). Immune precipitation was used to identify which glycoprotein complexes were sufficient for binding TLR2; gH/gL and gB could each bind TLR2 while gD was not able to bind.

Deletion or mutation of a pathogen sensor, e.g., a TLR, can have significant effects on the ability of a host to mount a proper immune response to pathogen infection. Two reports have identified defects in TLR3 expression/function that are critical to the development of HSV encephalitis (Zhang et al., 2007; Guo et al., 2011). Two patients suffering from HSV encephalitis were determined to have identical mutations in TLR3. The mutation (*cytosine* → thymine) at nucleotide 1660 resulted in an amino acid substitution (proline → serine) at position 554. Mutation at this position is thought to affect binding of the cognate ligand, dsRNA, to TLR3. Fibroblasts harvested from each patient showed a decreased ability to respond to the dsRNA mimic polyinosine-polycytidylic acid [poly(I:C)] (Zhang et al., 2007). IFN-β and IL-6 expression were both decreased in response to poly(I:C) in cells isolated from TLR3 deficient patients compared to cells isolated from healthy donors not harboring the mutation (Zhang et al., 2007). NF-κB and IRF3 expression were also impaired when compared to fibroblasts from healthy donors. Interestingly, however, PBMCs isolated from these patients showed normal production of IFN-α when challenged with a wide array of viruses, both RNA and DNA viruses (Zhang et al., 2007). The defect in immune response seemed to be specific to only HSV-1 and vesicular stomatitis virus (VSV) in fibroblasts. Additionally, five patients carrying the mutation did not develop HSV encephalitis. These last two points indicate the need for more studies into the role of TLRs in disease progression and the need for a clearer understanding of the possible redundancy within the TLR family.

Herpes simplex virus (HSV-2) was one of the first herpesviruses shown to activate TLR signaling. Infection of mouse bone marrow cells, which contain a high percentage of pDCs, with both live HSV-2 and UV-inactivated HSV-2 showed significantly increased IFN-α production (Lund et al., 2003). It was also determined that the adapter protein MyD88 was required for IFN-α production. HSV-2 DNA was recognized by TLR9 and an intact endocytic pathway was required for TLR9 mediated IFN-α production (Lund et al., 2003).

Another recent report has shown that HSV-2 can activate both TLR4 and TLR9 signaling in human cervical epithelial cells (HCE) (Li et al., 2009). *In vitro* infection of human cervical epithelium with HSV-2 resulted in increased levels of TLR4 and TLR9 mRNA and a concomitant increase in protein expression for each TLR. NF-κB was also induced as a result of infection with HSV-2 and its expression could be augmented with co-transfection of a TLR4 expression construct. IL-6 and IFN-β levels were also increased following HSV-2 infection of HCE cells (Li et al., 2009).

#### HSV encoded antagonists of TLR signaling and interferon activation

HSV encodes several proteins that can inhibit downstream signaling following TLR activation. The immediate early protein, ICP0, encoded by HSV-1 induces the degradation of MyD88 and its adaptor protein, TIRAP/MAL (Van Lint et al., 2010). Another HSV-1 encoded protein, the virion host shut-off protein (VHS) which has endonuclease activity, is thought to inhibit TLR3 signaling in conventional DCs since VHS deficient viruses could induce much higher pro-inflammatory cytokines from these cells (Cotter et al., 2010). The principal downstream target of TLR signaling is the induction of type I IFN through activation of IRFs. ICP0 is an E3 ubiquitin ligase that can either bind to IRF3 or degrade it and prevent its ability to activate IFN, or prevent the accumulation of IRF3 in the nucleus (Melroe et al., 2004, 2007; Paladino et al., 2010).

### Varicella zoster virus

Primary infection with varicella zoster virus (VZV) also known as human herpesvirus 3 (HHV-3) results in varicella, commonly known as chicken pox [reviewed in Gershon et al. (2010)]. Once the initial infection has been cleared by the host immune system the virus enters a latent state in both neurons and spinal dorsal root ganglia. Upon reactivation VZV presents as herpes zoster, or shingles, this infection is usually cleared by the host; however, complications such as post-herpetic neuralgia can arise, most often in immune compromised individuals (Gershon et al., 2010). The virus can re-enter latency following the clearance of shingles and continue to persist in the host. IFN production in response to VZV infection has been observed, as has inflammatory cytokine production (Arvin et al., 1986; Torigo et al., 2000). Both of these characteristics of VZV infection are hallmarks of TLR activation.

In 2005, Wang et al. described activation of TLR2 upon infection of monocytes and macrophage with VZV. The response was characterized by induction of the inflammatory cytokine IL-6 mediated by activated NF-κB (Wang et al., 2005b). Specific inhibition of TLR2 using siRNA resulted in decreased levels of IL-6 suggesting a specific upregulation of TLR2 on monocytes and macrophage subsequent to VZV infection. UV-inactivated VZV also led to increased IL-6 production.

Primary infection with VZV activates TLR9 in pDCs leading to increased IFN-α production (Yu et al., 2011). Purified pDCs were infected with live or UV-inactivated VZV and IFN-α levels were measured by ELISA. pDCs infected with live VZV showed strong induction of IFN-α, while pDCs infected with UV-VZV showed reduced levels of IFN-α. It was determined by treating pDCs with specific inhibitors of TLR9 that a majority of the IFN-α response was due to activation of TLR9 signaling (Yu et al., 2011). The reduced levels of IFN-α observed following infection with UV-VZV might occur through a TLR9-independent mechanism of IFN-α induction, perhaps through the RNA dependent protein kinase (PKR), which was activated following VZV infection and played a role in IFN-α production (Yu et al., 2011).

There is recent evidence that DCs infected with a clinical isolate of VZV (JoSt) respond differently to TLR2 stimulation than DCs infected with the vaccine strain of VZV (V-Oka) (Gutzeit et al., 2010). DCs infected with the JoSt strain of VZV and stimulated with lipoteichoic acid (LTA), a TLR2 agonist, secreted dramatically less IL-12 than DCs infected with the vaccine strain and challenged with the same TLR2 agonist (Gutzeit et al., 2010). IL-12 secretion from DCs is critical for the development of adaptive immune responses to infection. Therefore, the fact that virulent VZV (JoSt) blocks this secretion suggests a mechanism through which the virus is able to evade the adaptive immune response. It also highlights why the vaccine strain is effective in mounting an antiviral response (Gutzeit et al., 2010).

#### VZV encoded antagonists of TLR signaling and interferon activation

Currently, roles for two VZV viral proteins have been identified. The VZV kinase, Orf47p, has been shown to induce an atypical phosphorylation event on IRF3 that is inhibitory and prevents IRF3 homodimerization and induction of type I IFN (Vandevenne et al., 2011). Another viral protein, IE62, was shown to prevent TBK1-mediated activation of IFN-β expression. IE62 also inhibited IRF3 function by blocking phosphorylation of IRF3 at sites that are needed for activation (Sen et al., 2010). Inhibition by these two viral proteins would significantly affect the ability of the host to mount TLR driven immune responses following virus infection.

## β-Herpesviruses

### Human cytomegalovirus

In 2003, human cytomegalovirus (HCMV), also known as human herpesvirus 5 (HHV-5) was the first herpesvirus shown to trigger TLR mediated signaling events (Compton et al., 2003). CMV activates TLR2, leading to NF-κB-mediated upregulation of inflammatory cytokines. Both IL-6 and IL-8 were increased following infection of human PBMCs with CMV. PBMCs infected with UV-inactivated CMV also showed increased IL-6 and IL-8 secretion indicating no requirement for replication competent viral particles to stimulate this response (Compton et al., 2003). HEK293 cells stably expressing either TLR2 or TLR4 were infected with CMV and analyzed for production of IL-8 (Compton et al., 2003). Only infection of TLR2 expressing cells resulted in increased IL-8 secretion. It was also determined that TLR2 activation of inflammatory cytokines is mediated through NF-κB activation. Additionally, thioglycolate-elicited peritoneal macrophages (PECs) were isolated from wild type, TLR4^−/−^, and TLR2^−/−^ mice and infected with CMV. PECs from TLR4^−/−^ mice showed normal IL-6 production in response to CMV infection, while PECs from TLR2^−/−^ secreted no detectable IL-6. PECs from both knockout mice responded normally to their cognate ligands (zymosan/TLR2 and LPS/TLR4) (Compton et al., 2003). These results indicate that IL-6 upregulation following CMV infection of PECs is mediated specifically through TLR2, because even in the presence of functional TLR4 (TLR2^−/−^ mice) there was no detectable IL-6 in response to CMV infection (Compton et al., 2003).

In 2006, continued study into the activation of the innate immune response to CMV revealed that two viral proteins were responsible for TLR2 recognition, the glycoproteins gB and gH (Boehme et al., 2006). gB and gH are required for TLR2 recognition of CMV and both proteins co-immunoprecipitate with TLR1 and TLR2. Pre-treatment of UV-inactivated CMV particles with antibodies against gB and gH prior to infection of human fibroblasts resulted in a 40–50% reduction in secreted IL-6, confirming the importance of the recognition of gB and gH by TLR2 during CMV infection (Boehme et al., 2006).

Recently, HCMV infection has been shown to result in upregulation of TLR2, TLR3, and TLR9 in monocytes in the presence of the human monocyte scavenger receptor A type 1 (SR-A1) (Yew et al., 2010). TLR2, Lyn kinase and the p35 subunit of IL-12 were all upregulated within 10 min of HCMV infection in THP-1 monocytes. TLR3 and TLR9 levels were increased after 1 hr of HCMV infection (Yew et al., 2010). This is evidence of activation of multiple TLR pathways in a single cell. This group later showed that blocking Lyn kinase, which is associated with SR-A1, leads to inhibition of TLR9 signaling and shifts the response to a primarily TLR3 driven IFN-β response but also a non-canonical TLR3 driven NF-κB response (Yew and Harrison, 2011).

#### CMV encoded antagonists of interferon and chemokine induction

The immediate-early 2 gene product IE86 has been identified as an inhibitor of both IFN-β production and chemokine production. Initially, IE86 was identified as being able to block IFN-β production following both HCMV infection and Sendai virus infection (Taylor and Bresnahan, 2005). Soon thereafter the same lab determined that HCMV IE86 can also block chemokine induction, including IL-8, *CCL5, CCL3, and CCL8* after HCMV and Sendai virus infection (Taylor and Bresnahan, 2006b). Each of these chemokines can be induced following activation of TLR signaling. Lastly, a mechanism of action for IE86 was discovered, possibly explaining the ability of IE86 to have such a dramatic effect on the levels of immune response genes following virus infection. IE86 inhibits NF-κB transcriptional activation by preventing binding of NF-κB to DNA, specifically to the IFN-β promoter (Taylor and Bresnahan, 2006a). IE86 was also shown to be critical for TNF-α driven NF-κB transcription of both *CCL5* and IL-8 (Taylor and Bresnahan, 2006a).

### Human herpesvirus-6 (6A and B)

Human herpesvirus-6 is a ubiquitous human virus infecting over 90% of the world's population (Chi et al., 2012). The most common outcome of HHV-6 infection is *exanthem subitmum*, also known as “roseola.” HHV-6 was initially isolated from the blood of patients with lymphoproliferative disorders, including AIDS (Salahuddin et al., 1986).

Recently a role for TLR activation has been uncovered following infection of CD4+ T cells with HHV-6A (GS strain) (Chi et al., 2012). This study revealed that HHV-6A infection of CD4+ T cells resulted in the upregulation of TLR9 mRNA and protein levels. HHV-6A infection also led to activation of JNK and MAPK signaling pathways, including increased levels of phosphorylated JNK (Chi et al., 2012). Increased secretion of IL-6 and TNF-α was also secreted following HHV-6A infection.

A second recent report suggests that upon stimulation with TLR ligands, cells infected with HHV-6B show decreased levels of cytokine production in response to ligand treatment (Murakami et al., 2010). In this study HHV-6B infected dendritic cells were stimulated with ligands against TLR3 [poly(I:C)], TLR4 (LPS), and TLR7 (imidazoquinoline). In each case treatment with the TLR ligand resulted in decreased cytokine production when compared to mock-infected cells treated with the same dose of TLR ligand (Murakami et al., 2010). No mechanism for this apparent inhibition of cytokine production as a result of HHV-6B infection was proposed by the authors, however, it is an interesting finding that suggests an inhibitory role for HHV-6B during latency.

## γ-Herpesviruses

### Epstein-barr virus

Epstein-Barr virus (EBV), also known as human herpesvirus 4 (HHV-4), is one of the most ubiquitous pathogens in the human population, infecting over 90% of the world's population (Cesarman, 2011). EBV infection can lead to multiple outcomes, ranging from infectious mononucleosis to cancer, including Burkitt's lymphoma and nasopharyngeal carcinoma (Cesarman, 2011). Several reports have indicated a role for TLR signaling upon primary EBV infection in multiple cell lines. In 2007, three different TLRs activated by EBV infection in three distinct cell types were identified. The initial report identifying a role for TLR signaling during EBV infection found that TLR2 was activated in both human monocytes and HEK-293 cells stably expressing TLR2 (Gaudreault et al., 2007). TLR2 activation led to increased NF-κB expression and secretion of the chemokine *CCL2*. Activation of TLR2 was confirmed by pre-treating cells with blocking antibodies to TLR2 prior to EBV infection. NF-κB levels were significantly decreased in cells pre-treated with blocking anti-TLR2 antibodies indicating TLR2 specific recognition in B cells. Infection of HEK293-TLR2 cells with UV-inactivated EBV and infection of TLR2 expressing cells pre-treated with phosphonoacetic acid (a viral DNA polymerase inhibitor) also led to increased NF-κB expression, indicating that TLR2 could recognize intact virions and that stimulation was not dependent on viral replication, only on binding of EBV to the cell surface (Gaudreault et al., 2007).

A second report in 2007 indicated that EBV infection of B cells, the natural reservoir for EBV, led to upregulation of TLR7 and enhanced B cell proliferation. This was observed for infection of B cells with both wild type EBV and UV-inactivated EBV (Martin et al., 2007). Additionally, induction of a dominant negative form of IRF5 was observed following EBV infection. This is evidence that not only can EBV activate these innate immune pathways but that it can also manipulate them. Activation of wild type IRF5 typically results in tumor suppressive and antiviral activities, however, EBV specific induction of a dominant negative IRF5 indicates that the virus is capable of inhibiting the anti-viral effects of cellular IRF5 (Martin et al., 2007).

In 2009 the EBV dUTPase (BLLF3) was shown to activate NF-κB specifically through TLR2 (Ariza et al., 2009). In both HEK293 cells stably expressing TLR2 and human monocyte derived macrophages, proinflammatory cytokine production (IL-6) and NF-κB activation could be inhibited by treatment of cells with blocking anti-TLR2 antibody (Ariza et al., 2009). This was the first report of TLR recognition of a nonstructural herpesvirus protein leading to proinflammatory cytokine production.

EBV infection of pDCs, a subset of DCs, that are recognized as the most prolific producers of type I IFN in response to virus infection, was shown to result in increased IFN-α production (Lim et al., 2007). This report used an *in vivo* humanized mouse model to show that mice reconstituted with human PBMCs enriched with pDCs and challenged with EBV showed increased survival over mice reconstituted with non-enriched PBMCs (Lim et al., 2007). The increased survival rate was attributed to TLR9 activation of pDCs and the subsequent upregulation of IFN-α. Activation of natural killer cells (NK) and IFN-γ producing T cells was also a result of the activated pDCs in the mice reconstituted with pDC enriched PBMCs. pDCs along with primary monocytes were also shown to respond to EBV infection via TLR9 (Fiola et al., 2010). This study showed that treatment of both monocytes and pDCs with the endosomal acidification inhibitor, chloroquine, led to decreased levels of secreted proinflammatory cytokines, e.g., IL-8 (Fiola et al., 2010). Inhibition of TLR9 via a TLR9-specific ODN compound also led to decreased cytokine secretion including IFN-α and IL-6, in addition to IL-8 (Fiola et al., 2010).

In addition to TLR9, EBV infection of pDCs has also been shown to activate TLR7 signaling. Quan et al. showed that primary infection of pDCs led to activation of TLR7 and TLR9 leading to increased IFN-α (Quan et al., 2010). Increased IFN-α was observed following infection with wild-type EBV and UV-inactivated virions. EBV DNA alone was not able to stimulate IFN-α production. Pre-treatment of pDCs with chloroquine led to decreased IFN-α in a dose dependent manner. This evidence, combined with the UV-inactivation data, indicated that replication is not required for TLR9 mediated IFN-α production. The authors also investigated whether EBV-encoded RNAs (EBERs), small RNAs produced during EBV latency, could stimulate IFN-α production from pDCs (Quan et al., 2010). pDCs transfected with EBERs showed increased IFN-α levels, and those levels could be inhibited with treatment with inhibitory oligonucleotides specific to TLR7. IFN-α levels were not changed in response to EBERs in the presence of TLR9 specific inhibitors, indicating a specificity for TLR7 (Quan et al., 2010).

Recently, B cells undergoing EBV lytic replication were also shown to stimulate TLR9 (Van Gent et al., 2011). B cells were infected with increasing amounts of EBV and levels of the activation marker CD54 were compared to cells treated with the TLR9 agonist, CpG. CD54 increased with increasing amounts of EBV similarly to treatment with CpG (Van Gent et al., 2011). All of the above studies indicate how widespread and varied TLR activation can be and that activation can occur through multiple TLRs depending on the cell type.

#### EBV encoded antagonists of TLR signaling and interferon activation

Several EBV proteins have been shown to play a specific role in TLR signaling. EBV encodes a tegument protein, LF2 that interacts with IRF7 and suppresses IRF7-mediated IFN-alpha production (Wu et al., 2009). Additionally, both EBV LMP1 and the EBV lytic protein BGLF5 have been shown to downregulate levels of TLR9 by inhibiting TLR9 transcription or inducing TLR9 RNA degradation, respectively (Fathallah et al., 2010; Van Gent et al., 2011).

### Kaposi's sarcoma-associated herpesvirus

Kaposi's sarcoma-associated herpesvirus (KSHV), also known as human herpesvirus 8 (HHV-8), is the etiological of Kaposi sarcoma and the primary cause of two B cell lymphoproliferative disorders, primary effusion lymphoma (PEL) and multicentric castleman's disease (MCD) (Chang et al., 1994; Ablashi et al., 2002). KSHV is also the leading cause of cancer in HIV infected individuals [reviewed in Henke-Gendo and Schulz (2004)]. KSHV encodes many proteins capable of manipulating the host immune system but prior to 2008 there was no published data on the activity of TLRs in response to primary KSHV infection or during the process of reactivation.

Our lab reported the first evidence for KSHV activation of TLR signaling showing that primary KSHV infection of both monocytic leukemia cells (THP-1) and primary human monocytes resulted in increased levels of TLR3 and subsequently increased IFN-β production (West and Damania, 2008). We also observed concomitant increases in several key inflammatory cytokines, including CXCL10 and IL-6. Knockdown of TLR3 using shRNA prior to KSHV infection resulted in decreased IFN-β indicating TLR3 is the primary responder to KSHV infection in monocytes (West and Damania, 2008). We also observed increased NF-κB expression following KSHV infection in HEK293 cells stably expressing TLR3 compared to normal HEK293 cells (West and Damania, 2008).

Endothelial cells are one of the cell types infected by KSHV. It was shown in 2008 that KSHV infection led to downregulation of TLR4 (Lagos et al., 2008). This study showed that two viral proteins contributed to the decreased levels of TLR4, vIRF1, and vGPCR. This was the first report of a virus targeting TLR4 for immune evasion purposes (Lagos et al., 2008).

In 2009, our lab showed that TLRs can also play a critical role during reactivation of KSHV from latency (Gregory et al., 2009). We provided the first evidence that TLR stimulation can lead directly to reactivation of KSHV from latency. Treatment of KSHV latently infected B cell lines with the cognate agonists for TLR7/8 resulted in reactivation of KSHV, as observed by lytic viral gene and protein expression (Gregory et al., 2009). In addition to synthetic ligands we also showed that exposure of KSHV latently infected B cells to secondary infection with the known TLR7 agonist, VSV, led to significant reactivation of KSHV. This demonstrated for the first time that TLR activation, via a biologically relevant stimulus, could result in reactivation of KSHV (Gregory et al., 2009).

As described above for EBV and HSV, pDCs are key players in the innate immune response, particularly in the establishment of the antiviral state via production of type I IFN. pDCs have also been shown to be activated in response to KSHV infection and that activation leads directly to significant increases in IFN-α production (West et al., 2011). Increased expression of activation markers CD83 and CD86 was also observed following KSHV infection of pDCs. It was determined that increased IFN-α secretion was a direct result of TLR9 activation following KSHV infection (West et al., 2011). pDCs treated with inhibitory ODNs prior to KSHV infection showed decreased levels of IFN-α secretion compared with pDCs pre-treated with control ODNs (West et al., 2011). There was some residual IFN-α secretion that could be attributed to TLR7 activation, however, that possibility was not investigated. Interestingly, unlike many of the previous studies involving herpesvirus activation of TLR signaling in pDCs, infection with UV-inactivated KSHV did not result in upregulation of IFN-α, indicating that TLR9 actually recognizes KSHV DNA upon infection of pDCs.

#### KSHV encoded antagonists of TLR signaling and interferon activation

Several KSHV proteins have been identified as inhibitors of TLR signaling. Two proteins encoded by KSHV, vIRF1, and vGPCR, have been shown to downregulate expression of TLR4 (Lagos et al., 2008). KSHV encodes four different viral IRFs (vIRFs) which show some similarity to cellular IRFs. Three of these vIRFs can inhibit the action of cellular IRFs by interacting with them and preventing their transcriptional function and activation of IFN-α and IFN-β [reviewed in Jacobs and Damania (2011)]. Another KSHV encoded protein, Orf45, inhibits type I IFN production by preventing IRF7 phosphorylation and nuclear accumulation (Zhu et al., 2002, 2010). The immediate early protein, KSHV Rta/Orf50, has been shown to promote IRF7 ubiquitination and degradation and also induce the degradation of the TLR3 adaptor, TRIF (Wang et al., 2005a; Yu et al., 2005; Yu and Hayward, 2010; Ahmad et al., 2011). KSHV latency associated nuclear antigen also inhibits expression of IFN-β activation by IRF3 (Cloutier and Flamand, 2010).

## Concluding remarks

Herpesviruses are renowned for their ability to modulate host immune responses upon infection in order to achieve latency. TLR recognition is the first step in pathogen sensing in the host and over the last 10 years understanding the role of TLR activation during virus infection has been a focus of investigation in the herpesvirus field and has expanded our knowledge as to how herpesvirus recognition occurs during primary infection. TLR signaling has also been implicated during reactivation of herpesviruses, a process essential for these viruses to maintain themselves in the host.

Defects in TLR expression in patients suffering from diseases caused directly by herpesvirus infection has also served to shed light on the role of TLR signaling during virus infection. The inability of these patients to mount proper immune responses to virus infection highlights the importance of these signaling pathways during infection and eventual disease progression. Continued investigation into TLR function in patients suffering from herpesvirus related disease would provide important *in vivo* data that could be used to help discover new targets for treatment of these viral infections. Already several clinical trials have been initiated to determine whether TLR agonists could be used as adjuvants in potential cancer vaccines [reviewed in Gregory et al. (2011)].

Ongoing investigation into virally encoded inhibitors of TLR signaling will be critical for discovering new possible treatment options. At this point there are only a limited number of herpesvirus proteins that disrupt TLR signaling, however, based on the number of known immune modulatory proteins encoded by herpesviruses [reviewed in Paludan et al. (2011)] it is likely that there are several uncharacterized viral proteins that play a role in the manipulation of TLR signaling. Continuing to understand the contribution of TLR signaling during herpesvirus infection, and the virus counter response to TLR signaling, will help in designing better vaccine candidates and therapeutics against this family of viruses.

### Conflict of interest statement

The authors declare that the research was conducted in the absence of any commercial or financial relationships that could be construed as a potential conflict of interest.
